RETRACTED

# The Nursing Effect of PRECEDE Management on Occupational Exposure to Surgical Smoke: Based on a Randomized Controlled Study

**DOI:** 10.1155/2022/8610517

**Published:** 2022-05-20

**Authors:** Hong Ye, Dan Xin, Xuefei Hu

**Affiliations:** ^1^Wuhan No.1 Hospital Operating Room, China; ^2^Wuhan No.1 Hospital Intervention Department, China

## Abstract

**Background:**

Occupational exposure seriously threatens the physical and mental health of professionals and has become an important public health problem. In clinical medical and nursing work, medical staff, especially nursing staff, are faced with the status quo of occupational exposure with high risk, serious harm, and severe situation. Therefore, a sound management system must be established to control the occupational exposure of nurses.

**Aims:**

According to the PRECEDE management model, evaluate the operating room nurses' knowledge, belief, and behavior scores on the protection of surgical smoke, understand their awareness of surgical smoke and the current status of protection, improve the mastery rate and protection compliance of surgical smoke-related knowledge in the operating room, reduce the harm of surgical smoke to the human body, and provide a basis for smoke protection.*Materials and methods*. 125 doctors working in the operating room of our hospital were selected as the control group of this study, and 112 nonsmoke-exposed nurses working in the operating room of our hospital were selected as the observation group. The nurses' knowledge-belief behavior scores and self-evaluation scores of smoke influence were counted before and after the intervention in the operating room. SPSS25.0 was used to process the data. Tests and repeated measures analysis of variance were used to compare the effects before and after intervention.

**Results:**

After one month of intervention, the knowledge scores of nurses in the operating room on the protection of surgical smoke increased significantly, and the difference was significant (*P* < 0.05); the scores of related concepts, physical properties, chemical properties, and authoritative protection standards increased significantly (*P* < 0.05). There was no significant increase in the scores of smoke hazards (*P* > 0.05); the attitude of smoke protection increased significantly, which was statistically significant (*P* < 0.05); and the behavior compliance of smoke protection was significantly increased, which was statistically significant (*P* < 0.05). After one month of intervention, the self-evaluation score of smoke effect of operating room nurses decreased significantly, and the difference was statistically significant (*P* < 0.05). The data was analyzed by repeated measure analysis of variance. The knowledge of surgical smoke (*F* = 65.570, *P* < 0.001), attitude (*F* = 78.307, *P* < 0.001), and behavior (*F* = 403.015, *P* < 0.001) scores gradually increased. The observation group's total cholesterol, low-density lipoprotein cholesterol, and the proportion of low-density lipoprotein cholesterol were higher than that of the control group, and the proportion of high-density lipoprotein cholesterol was lower than that of the control group. The difference was statistically significant *P* < 0.05.

RETRACTED

**Conclusion:**

After the intervention of operating room nurses under the guidance of PRECEDE management mode, the theoretical knowledge of operating room nurses is effectively improved, the operations are standardized, the self-evaluation scores of smoke influence are reduced, and the safety level of operating room is improved. More importantly, the health of nursing staff is fully guaranteed.

## 1. Introduction

The operating room is a fast-paced, independent closed, and high-risk special department. It is a key place for performing operations and saving lives [1, 2]. The ultrasonic knife, high-frequency electrosurgical knife, and laser knife used in surgery are used by doctors in modern surgical operations because of their fast hemostasis speed and good effect. However, while using these instruments and equipment to benefit the majority of patients, products such as smoke, gas, and particles will also be produced, which not only blur the surgical field of vision but also contain various toxic substances, which cause a certain degree of harm to the operating room staff. [3].

Surgical smoke is harmful to the health of occupationally exposed people, but due to the low exposure dose, the effect cannot be expressed quickly. In order to clarify whether it has a specific and monitorable impact on the human body, refer to other smoke exposure hazard research indicators to initially discuss the impact of surgical smoke on occupations and the health effects of exposed populations [4]. In order to lay the foundation for further targeted research and increase the exposure of the exposed population to hazards, it is very necessary. At the same time, the awareness and basic knowledge of the surgical smoke exposure of the population exposed to surgical smoke is the first step to take effective protective measures. It is necessary to understand it to further develop training programs [5]. However, at present, the majority of medical staff do not pay enough attention to the smoke generated by the operation, and the operating room is full of various risk factors. Among them, the surgical smoke, as a kind of risk factor, has harmed the health of the medical staff in the operating room [6]. Therefore, it is necessary to systematically study the hazards of surgical smoke and take relevant measures to improve their protection awareness and reduce occupational hazards [7]. The PRECEDE management was developed by Lawrence Green and refers to the development of health education programs that rely on information collection and judgment and analysis. Three environmental assessment factors were included in the process, that is, tendency factor, enabler factor, and intensification factor. PRECEDE management emphasizes the objective evaluation of predisposing factors, contributing factors, and reinforcing factors that influence health behaviors in the design of intervention programs and the formulation of measures to overcome them with each of these parts. PRECEDE evaluates the research object in all aspects, finds out the causes and characteristics of certain behaviors, formulates intervention plans and measures, strengthens the research object's theoretical level of disease or harm, promotes changes in their behavior, and evaluates the effect [8]. Many research scholars at home and abroad have applied the PRECEDE management model to the health education of patients, including health education for cardiovascular disease patients, health education for pregnant women, and health education for diabetes patients, chronic disease patients, and the elderly in the community [9]. Based on this, in the nursing effect of our hospital PRECEDE management on occupational exposure to surgical smoke, based on a randomized controlled study, some exploration has been carried out, and the current research results are reported as follows.

RETRACTED

## 2. Material and Methods

### 2.1. Research Object

Before the start of the study, nurses and family members were informed and signed an informed consent. 125 doctors who worked in the operating room of our hospital from January 2019 to December 2021 were selected as the control group of this study and selected in our hospital during the same period. 112 nonsmoke-exposed nurses working in the operating room were in the observation group.

### 2.2. Exclusion Criteria

Inclusion criteria were as follows: (i) no history of chronic diseases, no family history of hyperlipidemia, hypertension, high hemoglobin, or anemia, no X-ray exposure within six months, and no recent history of viral infection; (ii) because the time limit of surgical smoke exposure is retrospectively recorded and exposed, the time limit is different, and it is difficult to accurately count the specific time. Therefore, the observation group selected medical staff who were exposed to surgical smoke for more than 5 years, the number of contacts per week >10 times, and each contact time >10 min.; and (iii) nurses who are registered and on-the-job nurses in the operating room who agree to fill out the questionnaire.

RETRACTED

### 2.3. Exclusion Criteria

Exclusion criteria were as follows: (i) there are factories that emit toxic and hazardous substances around the place of residence, recent blood donation history, pregnant, or lactating women; (ii) training personnel, interns, and nurses who ask for leave or go out, nurses who refuse to fill in the questionnaire, and nurses that have diseases that can impact the test; and (iii) patients with severe miscarriage and mental disorders.

## 3. Nursing Intervention Methods

### 3.1. Tendency Factor Intervention

In special lectures organized by the department (the definition and generation of surgical smoke in the first week, the hazards of surgical smoke in the second week, the protection standards of international authoritative organizations and the small inventions for filtering surgical smoke in the third week, and the prevention of surgical smoke in the fourth week Measures), we issue educational materials on smoke protection, consult relevant domestic and foreign materials, summarize and print them (including the definition of surgical smoke, sources, ingredients, effects on the human body, protective measures, and authoritative protection standards) and conduct surgical smoke related theories training, including definitions, sources, ingredients, and hazards to the human body, effective protective measures and international authoritative organization protection standards, etc. The lectures are conducted in rotation by the head nurse of the department and the head of the professional group. The lectures are held in the morning meeting every week, and each time is 15-30 minutes. The time, place, and content of each lecture will be informed by the leader of the professional group responsible for teaching, and the nurses in the operating room will be urged to participate.

### 3.2. Facilitating Factor Intervention

The department is equipped with protective equipment and smoke filtering devices and equipment, and we purchase high-filter masks (N95 or NI00 masks), smoke filters, and negative pressure suction devices with good clinical effects and use of improved ones during the operation. Antismoke devices, such as integrated smoking equipment, and special smoke exhaust pipes for laparoscopic surgery [38] were modified from blood transfusion sets. (Before the operation, the nurse cut the blood transfusion set on the operating table to remove the cork and puncture device for the vein. The needle and the mofe dropper become a smoke exhaust tube formed by a catheter, regulator, and cone. During the operation, connect the cone of the smoke exhaust tube to the observation hole and the side hole of the operating hole, and in the other end, connect the suction device and seal it with a sterile infusion patch). A protective smoke management group is formed, consisting of 1 deputy head nurse, 2 senior nurses, and 1 nurse of the endoscopy specialist group; supervise the implementation of protective behaviors among nurses.

RETRACTED

### 3.3. Strengthen Factor Intervention

Establish WeChat groups or QQ groups, the group owners regularly push smoke theoretical knowledge and hazards and protective measures, and the members of the group communicate with each other, share experiences, brainstorm ideas, and promote innovation. Regularly carry out and organize training and business learning for surgical smoke protection. In each operating room posted a smoke protection management form, which was filled out by the roving nurses and equipment nurses. The management team members regularly checked the completion of the plan and gave feedback and gradually identified and dealt with common problems that appeared.

### 3.4. Observation Indicators

Surgical Smoke Knowledge Questionnaire [10] has 20 items, the content is smoke concept (2 items), production (1 item), composition (1 item), physical properties (3 items), chemical properties (7 items), hazards (3 items)), and authoritative protection standards (3 items). Answer with judgement “√” and “×”, 1 point is awarded for correct answers, and no points are scored for incorrect answers. The score range is 0-20. The higher the score, the better the knowledge and theory of surgical smoke. There are 16 items in the Surgical Smoke Protection Attitudes Questionnaire, using the Likert Scale 5-level scoring method: options include “strongly disagree, disagree, neutral, agree, and strongly agree,” and each score is “1, 2, 3, 4, and 5,” the positive point of view is scored forward, and vice versa, and the score range is 16-80. There are 16 items in the protective surgical smoke behavior questionnaire, and the 5-level scoring method of the Likert scale is also used. The options include “cannot do it at all, occasionally do it, about half do it, most do it, completely do it,” the scores are “1, 2, 3, 4, and 5,” and the score range is 16-80. The higher the score, the more standardized its safe operation.

### 3.5. Statistical Analysis

We use Epidata to enter all the data and then use SPSS 25.0 to statistically process the data. The data needs to be entered into a computer database by a second person to ensure the completeness and accuracy of the data. *χ*^2^ test is used to express the count data as a percentage (%). For each parameter, data is mentioned as mean ± SD and statistically analyzed by employing one-way ANOVA followed Tukey's multiple comparisons post hoc test. *P* < 0.05 is considered as statistically significant.

RETRACTED

## 4. Results

### 4.1. General Information Comparison

The average age, body mass index, average monthly income, professional title, and other general data of the two groups of nurses were not significantly different by *t* test (*P* > 0.05), see Table 1.

### 4.2. Comparison of Knowledge-Faith-Action Scores

According to the test standard of *α* = 0.05, in the operating room nurses' theoretical knowledge score (*t* = 3.726, *P* < 0.05), protective attitude score (*t* = 2.303, *P* < 0.05), protective behavior score (*t* = 14.29, *P* < 0.05) before and after the intervention (*t* = 14.29, *P* < 0.05) compared with the significant increase, the result is statistically significant; the smoke impact score before and after the intervention is significantly reduced, and the result is statistically significant (*t* = 1.833, *P* < 0.05), see Figure 1.

### 4.3. Comparison of Nurses' Knowledge Scores in Operating Room

According to the test standard of*α* = 0.05, in the concept score before and after intervention (*t* = 3.869,*P* < 0.05), physical property score (*t* = 5.296,*P* < 0.05), chemical property score (*t* = 3.687,*P* < 0.05), and international authority, the organization protection standard score (*t* =3.687, *P* <0.05) is significantly higher than that, and it is statistically significant; according to the test standard of *α* = 0.05, H0 is not rejected, and it cannot be considered that the hazard score before and after intervention has changed significantly, and the result is not statistically significant. Significance (*t* = 0.011, *P* > 0.05), see Figure 2.

### 4.4. Comparison of Blood Test Indicators

The observation group TC and low-density lipoprotein cholesterol were higher than the control group, and the observation group TG and HDL-C were lower than the control group, but the difference was not statistically significant (*P* > 0.05). The hemoglobin and RBC specific product of the observation group were higher than the control group, the difference was statistically significant (*P* < 0.05); the RBC count and WBC count were higher than the control group, the absolute value of PLT count and lymphocytes was lower than the control group, but the difference was not statistically significant. *P* > 0.05was statistically significant, see Figures 3 and 4.

## 5. Discussion

Operating room nurses' poor awareness and protection of surgical smoke may be related to factors such as high work intensity, neglect of the harm caused by surgical smoke to the human body, and inadequate publicity of smoke hazards and occupational protection education in the department [11]. Smoke contains active bacteria and viruses, irritating ingredients, carcinogens, and tiny harmful particles, which can cause various chronic adverse reactions in the human body, lung damage, tumor cell planting and metastasis, and bacterial virus transmission, which can cause fatigue in the human body, throat pain, conjunctival congestion, nausea and vomiting, and other symptoms [12–14]. The PRECEDE management mode is used to intervene the standard prevention knowledge and behavior of operating room nurse, which improves the theoretical awareness and behavior implementation rate of operating room nurse, and reduces the incidence of occupational exposure of operating room nurse [15, 16].

RETRACTED

Under the guidance of the PRECEDE management model, this research trains operating room nurses and uses a variety of teaching methods to keep them abreast of the latest developments in smog at home and abroad, the international authoritative organization's guidelines for the protection of surgical smoke, and the concept, source, composition, and composition of surgical smoke [17–19], as well as theories of physical and chemical properties that harm to the human body. The results of repeated measure analysis of variance showed that the theoretical performance of operating room nurses on surgical smoke after the intervention was significantly higher than before the intervention, indicating that the PRECEDE management model promotes the operating room nurses to master the theory of surgical smoke [17, 20–22]. The operating room nurses' attitude toward operating smoke was significantly higher than that before the intervention, indicating that the training under the guidance of PRECEDE management model strengthened the operating room nurses' awareness of protection [23–25]. Therefore, improving the awareness and attitude of protection and correctly understanding the hazards of surgical smoke are the focus of promoting safe operation of operating room nurses, reducing occupational hazards, and ensuring the health of operating room staff. Moreover, the implementation of PRECEDE management model obviously promotes the theoretical level of nurses in the operating room and reduces the smoke effects on health [26–29].

Smoke reduces serum HDL levels and raises cholesterol levels in passive smokers. Cholesterol, especially low-density lipoprotein cholesterol levels, are positively correlated with the incidence of atherosclerosis and coronary heart disease, which leads to an increased risk of atherosclerosis and coronary heart disease in exposed populations. In particular, smoking, as a major risk factor for coronary atherosclerosis, has significantly increased the incidence and mortality of coronary heart disease, which should be given enough attention. The results of the study showed that on the basis of no difference in other influencing factors of blood lipids, the proportions of total cholesterol, low-density lipoprotein cholesterol, and low-density lipoprotein cholesterol in the observation group were higher than those in the control group, and the proportion of high-density lipoprotein cholesterol was lower than that in the control group. Other smoke studies have also shown similarities results [30, 31].

RETRACTED

The concentration of acrylonitrile and hydrogen cyanide in the surgical smoke in this study is relatively high and easily absorbed. The cyanide and hydrogen cyanide released after acrylonitrile are absorbed and inhibit respiratory enzymes, causing mild hypoxia in the body. The high concentration of surgical smoke leads to carboxyhemoglobin and methemoglobin increased, and the blood's oxygen-carrying capacity decreased in the exposed population. Long-term and continuous mild hypoxia will increase the secretion of erythropoietin from renal tubular interstitial cells, enhance the hematopoietic capacity of bone marrow, and lead to a compensatory increase in hemoglobin. The study found that hemoglobin and hematocrit of the observation group were higher than those of the control group [32–34]. This study used blood test items to initially understand the impact of surgical smoke on the health of people exposed to fog but did not analyze its impact on the body's immune function, genotoxicity, and lipid peroxidation damage at the molecular level. And this study is a cross-sectional study which has limitations also. Surgical smoke is a source of occupational exposure. Although there is no obvious source of industrial occupational exposure, in order to ensure the occupational safety of the exposed population, it is necessary to cooperate with the investigation of the current situation of surgical smoke pollution to follow up a larger sample for long-term follow-up and further research.

## 6. Conclusion

In summary, after the intervention of the PRECEDE management mode by the operating room nurses, the theoretical knowledge and attitude level of the operating room nurses have been effectively improved, the safety level of the operating room has been improved, the health of the nursing staff has been effectively protected, and the implementation of smoke protection measures has been strengthened, thereby improving the nurse's blood lipid level and reducing the harm caused by smoke to the human body.

RETRACTED

## Figures and Tables

**Figure 1:** Comparison of knowledge-belief-action scores according to the test standard of *α* = 0.05, the theoretical knowledge score (a), protective attitude score (b), and protective behavior score (c) of nurses in the operating room before and after intervention compared with a significant increase, and the smoke impact score (d) before and after the intervention was significantly reduced. Values are presented as mean ± SD and analyzed by one-way ANOVA.

**Figure 2:** Comparison of nurse knowledge scores in operating room. The concept score (a), physical property score (b), and chemical property score (c) before and after the intervention are significantly improved compared to the protection standard score of the international authoritative organization (d). However, the hazard scores before and after intervention (e) did not change significantly. Values are presented as mean ± SD and analyzed by one-way ANOVA.

**Figure 3:** TC and LDL cholesterol in the observation group are higher than those in the control group, and TG and HDL-C in the observation group are lower than those in the control group. The hemoglobin and hematocrit of the observation group were higher than those of the control group. Values are presented as mean ± SD and analyzed by one-way ANOVA.

**Figure 4:** RBC count and WBC count are higher than the control group, and PLT count and lymphocyte absolute value are lower than the control group. The RBC count and WBC count are higher than the control group, and the PLT count and the absolute value of lymphocytes are lower than the control group. Values are presented as mean ± SD and analyzed by one-way ANOVA.

**Table 1:** Comparison of general information between the two groups ([$\bar{x}\pm s$]).

Group	Average age (years)	Body mass index (kg/m^2^)	Average monthly income (thousand yuan)	Job title		
				Elementary	Intermediate	Advanced
Control group (*n* = 125)	37.23 ± 10.46	26.59 ± 3.09	6.86 ± 1.32	29	66	30
Observation group (*n* = 112)	36.13 ± 8.61	26.60 ± 3.10	6.87 ± 1.31	25	67	20
*t*	0.351	-0.025	-0.058	1.596		
*P*	0.726	0.980	0.953	0.450		

## Data Availability

No data were used to support this study.
